# Intelligent Physical Training Data Processing Based on Wearable Devices

**DOI:** 10.1155/2022/1207457

**Published:** 2022-05-20

**Authors:** Xuguang Liu

**Affiliations:** Nanjing University of Information Science and Technology, Nanjing 210044, China

## Abstract

Intelligent processing of physical training data based on wearable devices is conducive to improving the efficiency and rationality of physical training. The current data processing methods cannot effectively extract the features contained in the data, resulting in low accuracy in tasks such as classification. This paper proposes an intelligent processing method for sports training data based on statistical methods and deep learning methods. First, the original data are preprocessed by some statistical methods to obtain the original feature vector. Then, the autoencoder model is used to extract the high-level hidden features in the original data. Finally, we input the extracted feature vector into a designed convolutional neural network classification model and generate the final classification result. Evaluation on the open Human Activity Recognition Using Smartphones Dataset shows that our proposed method achieves the best results compared with current methods.

## 1. Introduction

Physical training is a basic means of physical and intellectual activities. According to the laws of human growth and development, skill formation, and function improvement, it can promote the all-round development of human beings, improve physical fitness and athletic ability, and is an important way to improve lifestyle and improve physical fitness [1]. It is a meaningful social activity for quality of life. The scale and level of sports development have become an important symbol for measuring the development and progress of a country and society, and it has also become an important means of diplomatic and cultural exchanges between countries. Physical education is a highly comprehensive subject, including humanities and sports sciences and sports social sciences.

Wearable computing technology [2] was the earliest innovative technology in the MIT Media Lab in the 1960s, and it is one of the most promising advanced technologies in the field of modern human-computer interaction. Wearable devices are smart devices that realize user interaction, human health monitoring, life entertainment, and other functions with the support of biosensing technology, wireless communication technology, and intelligent analysis software. It can achieve powerful functions through software support, data interaction, and cloud interaction, providing users with data monitoring support and decision-making assistance [3–6]. Wearable sensors are not only small in size and light in weight but also have the characteristics of low power consumption, simple operation, and wireless data transmission, which have always attracted the attention of a large number of researchers. Wearable devices have brought great changes to our lives, especially in sports training applications.

With the rapid development of computer science and artificial intelligence technology [7], especially the development of artificial intelligence theory and data mining processing technology, it provides a good theoretical and application basis for sports training data processing and advanced training methods based on wearable devices. With the continuous accumulation of sports training data, conventional statistical analysis techniques may be insufficient in the analysis of training data, and it is difficult to find a suitable model to describe the correlation between these data. The emergence of intelligent methods provides optimized methods for discovering scientific laws and correlations in large amounts of complex training data. The intelligent data analysis technology integrates multi-disciplinary technologies such as statistics, artificial intelligence, and information theory to conduct a comprehensive analysis of sports training indicators. Artificial intelligence (AI) is defined as the ability of a system to correctly interpret and learn from external data and to adapt flexibly to achieve specific goals and solve problems using the learning results. As a member of emerging technologies, artificial intelligence has already been applied in various fields such as speech recognition, image recognition, and unmanned driving. In a short period of time, artificial intelligence has moved from theory to practical application, providing more work assistance for humans, such as diagnosing diseases [8]. In addition, artificial intelligence can assist humans in decision analysis from a theoretical perspective. Machine learning is a subfield of artificial intelligence that provides decision analysis for people and contains numerous advanced algorithms. For example, neural network algorithms can be applied to solve the problem of optimizing sports training data processing [9].

For smart sports training data processing and classification models based on wearable devices, researchers have proposed many research methods, such as decision trees [10], K-nearest neighbors (KNN) [11], Bayesian methods [12], hidden Markov model (HMM) [13], and support vector machine (SVM) [14–16]. In the literature, various methods for dimensionality reduction of high-dimensional features of samples in classification and recognition tasks have been proposed [17–19]. The current research on action recognition based on wearable sensors still has many problems to be solved due to the difficulty of feature extraction and the diversity of action types.

In this paper, we propose an intelligent sports training data processing method based on a deep neural network. Firstly, the data are normalized and preprocessed, then the deep autoencoder is used to extract features from the data, and finally the extracted feature vectors are classified and identified, so as to provide reasonable adjustment and decision support for sports training.

The contribution of this paper can be summarized as follows:

1. We design a feature extraction method based on statistical methods, which can extract inherent features present in raw data from both time and frequency domains.
2. We design a feature extraction method based on autoencoders, which can obtain the high-level hidden features from the processed data.
3. We propose an intelligent physical training data processing method that can well recognize different types of motion poses, including walking, walking upstairs, walking downstairs, sitting, standing, and lying.

The rest of this paper is organized as follows.  Section 1 describes the studies about physical training data processing based on wearable devices.  Section 2 introduces the proposed method for physical data processing, including data preprocessing, feature extraction, and classification network.  Section 3 presents experimental studies and results to compare and demonstrate the state-of-the-art performance of the proposed model for physical training data processing.  Section 4 concludes the whole paper.

## 2. Method

In this section, we first introduce the details of the dataset used in our experiments, including preprocessing methods and steps. Then, we describe the designed model for feature extraction from the preprocessed data. Finally, we present the detailed steps for designing classification methods using deep neural network models.

The method proposed in this paper consists of three steps: (1) the original data are preprocessed by some statistical methods to obtain the original feature vector with dimension of 100; (2) the autoencoder model is used to extract the high-level hidden features in the original data to generate a feature vector with a dimension of 50; and (3) we design a convolutional neural network model, input the extracted feature vector, and generate the final classification result. The overall flowchart of the proposed model is shown in Figure 1. Each dashed box in the figure represents a processing step corresponding to the above. Below we will describe their detailed processing in detail.

### 2.1. Data Preprocessing

The raw data need to be converted into a digital matrix before they are used and subjected to subsequent classification and identification tasks. After preprocessing, we can obtain a 100-dimensional feature vector for each data sample, including calculation of mean values, kurtosis, variance, covariance, correlation coefficient, skewness, angular velocity, and acceleration of entropy and energy in the direction of *X*, *Y*, and *Z* axes, as shown in Table 1. These methods extract inherent features present in raw data from both time and frequency domains.

These methods have their own advantages. The mean is the sum of all data divided by the number of data points to express the average size of the dataset. The purpose of the variance is to express the degree of dispersion of data points in a dataset. Kurtosis is also known as the kurtosis coefficient. Intuitively, kurtosis reflects the sharpness of the peak. The kurtosis of a sample is a statistic compared to the normal distribution. If the kurtosis is greater than three, the peak shape is sharper and steeper than the normal distribution peak. Covariance expresses the error of the population of two variables, which is different from the variance that expresses the error of only one variable. If the trends of the two variables are consistent, that is, if one of them is greater than its own expected value and the other is also greater than its own expected value, then the covariance between the two variables is positive. If the trends of the two variables are opposite, that is, one of them is greater than its expected value and the other is less than its own expected value, then the covariance between the two variables is negative. Skewness is a measure of the direction and degree of skewness in the distribution of statistical data and is a numerical feature of the degree of asymmetry in the distribution of statistical data. The correlation coefficient is the specific measure that quantifies the strength of the linear relationship between two variables in a correlation analysis. The coefficient is what we symbolize with the *r* in a correlation report. Entropy generally refers to a measure of the state of certain material systems, the degree to which certain material system states may appear. It is also used by the social sciences as a metaphor for the degree of certain states of human society. The concept of entropy was originally used to describe “energy degradation” as one of the state parameters of matter, and it has a wide range of applications in thermodynamics. The essence of entropy is the “internal chaos” of a system. Energy is a measure of the degree to which the spatiotemporal distribution of mass may vary and is used to characterize the ability of a physical system to do work.

### 2.2. Feature Extraction

After computing the temporal and frequency-domain features of the data using statistical methods, we propose a feature extraction model that utilizes deep learning methods. That is, we utilize an autoencoder to perform feature extraction on the raw data.

Deep learning technology proposes a method for computers to automatically learn pattern features and integrates feature learning into the process of building models, thereby reducing the incompleteness caused by artificially designed features. A major advantage of deep learning over previous neural networks and other machine learning algorithms is its ability to infer new features from the limited set of features contained in the training set. That is, it will search and find other features that are related to known features. Deep learning techniques are new ways to extract useful signals from noisy data. Deep learning's ability to create features without being explicitly told means data scientists can save months of work by relying on these networks.

As a typical unsupervised deep learning model, autoencoders aim to learn abstract features of input samples by equating the expected output of the network with the input samples [20]. As a neural network used in unsupervised learning, the input and expected output of the autoencoder are unlabeled samples, and the output of the hidden layer is the abstract feature representation of the samples. Autoencoder first takes input samples, converts them into efficient abstract representations, and then outputs a reconstruction of the original samples. An autoencoder usually consists of two parts: an encoder and a decoder. The encoder maps high-dimensional input samples to low-dimensional abstract representations to achieve sample compression and dimensionality reduction; the decoder converts the abstract representations into desired outputs to reproduce the input samples. Different from the fully connected neural network, the connection method of autoencoder nodes can be fully connected or convolutional, but due to the unsupervised learning paradigm, the input and output of the autoencoder are unlabeled samples, and no label information is required. The purpose is to learn samples and extract abstract features. The traditional fully connected network adopts the supervised learning paradigm, and its output is the sample label, which aims to complete the mapping of features to labels.

In our method, first, we input the data into the encoder to extract high-level hidden features in the data through compression. Then, we pass the encoded data through the decoder to obtain the same size as the original data. Finally, the parameters of the autoencoder are continuously optimized by backpropagating the gradient of the difference between the decoded data and the original data, so as to obtain the extracted high-level hidden features. Its overall schematic diagram is shown in Figure 2.

The training process of the autoencoder includes two stages, including encoding and decoding. In the encoding process, the input samples are encoded to obtain the encoding layer. In the decoding process, the encoding layer is decoded to obtain the reconstruction of the input samples, and the reconstruction error is minimized by adjusting the network parameters to obtain the optimal abstract representation of the input features.

Assuming a given input sample *X* ∈ *R*^*n*×*m*^, the weight matrix between the encoding layer and the input layer is *W*, the encoding layer node bias is *b*_*e*_, the decoding layer bias is *b*_*d*_, and the node activation function is *f*(·); the autoencoder first passes linear mapping and nonlinear activation function to complete the encoding of the samples as follows:

(1) $$\begin{array}{c} \text{Hidden}=f\left(WX+b_{e}\right). \end{array}$$

Then, the decoder completes the decoding of the encoded features and obtains a reconstruction of the input sample $\hat{X}$. When given an encoding Hidden, $\hat{X}$ can also be seen as a prediction of *X* with the same dimensions as *X*. The decoding process is similar to the encoding process as shown below.

(2) $$\begin{array}{c} \hat{X}=f\left(W^{T}\text{Hidden}+b_{d}\right). \end{array}$$

After that, we can calculate the loss between the input data *X* and the decoded data $\hat{X}$ through the mean square error (MSE) loss function and cross-entropy (CE) loss function. Their definitions are shown as follows.

(3) $$\begin{array}{c} \text{MSE}\left(X,\hat{X}\right)=\frac{1}{2}\sum_{i=1}^{n}{\left\|{\hat{x}}_{i}-x_{i}\right\|}_{2}^{2}, \end{array}$$

(4) $$\begin{array}{c} \text{CE}\left(X,\hat{X}\right)=-\sum_{i=1}^{n}\left[x_{i}\log\left({\hat{x}}_{i}\right)+\left(1-x_{i}\right)\log\left(1-{\hat{x}}_{i}\right)\right], \end{array}$$

where **x**_*i*_ ∈ *X*, *i*=1,2,3,…, *n* and ${\hat{x}}_{i}\in \hat{X},i=1,2,3,\ldots ,n$. During training, our goal is to minimize the loss function, that is,

(5) $$\begin{array}{c} \text{arg}\underset{W,b}{\text{min}}\text{MSE}\left(X,\hat{X}\right),\\ \text{arg}\underset{W,b}{\text{min}}\text{CE}\left(X,\hat{X}\right). \end{array}$$

Then, we use the gradient descent algorithm to backpropagate the error to tune the network parameters and gradually minimize the reconstruction error function through iterative fine-tuning to learn key abstract features in the sample data. When the gradient descent algorithm is used, assuming that the learning rate is *η*, the connection weights and bias update formulas of the autoencoder are

(6) $$\begin{array}{c} W=W-\eta \frac{\partial J\left(W,b\right)}{\partial W}, \end{array}$$

(7) $$\begin{array}{c} b=b-\eta \frac{\partial J\left(W,b\right)}{\partial b}. \end{array}$$

By continuously training and optimizing the model parameters, an autoencoder with encoding ability will be finally obtained. With the trained autoencoder, we can use the encoder to take the original data as input to get the encoded feature vector. The algorithm flow is shown in Algorithm 1.

### 2.3. Classification

After the features are extracted by the autoencoder, we get a high-level feature vector of dimension 50 for each sample. We design a convolutional neural network model to classify and identify this feature vector, including walking, walking upstairs, walking downstairs, sitting, standing, and lying.

Convolutional neural network is an artificial neural network with multiple hidden layers specially designed by mimicking the structure of the biological cerebral cortex. Convolutional layers, pooling layers, and activation functions are the essential components of a convolutional neural network. The convolutional neural network reduces the complexity of the network model through three strategies of the local receptive field, weight sharing, and downsampling. At the same time, it is invariant to the degree of variation in the form of translation, rotation, and scaling. Therefore, it is widely used in image classification, target recognition, speech recognition, and other fields. In general, a common convolutional neural network consists of an input layer, a convolutional layer, an activation layer, a pooling layer, a fully connected layer, and a final output layer. Convolutional neural networks can effectively learn corresponding features from a large number of samples, avoiding the complex feature extraction process. The convolutional neural network has two characteristics of local perception and parameter sharing. Local perception is that the convolutional neural network proposes that each neuron does not need to perceive all the pixels in the image but only perceives the local pixels of the image. The local information is combined to obtain all the representation information of the image. The neural units of different layers are connected locally, that is, the neural units of each layer are only connected to some neural units of the previous layer. Each neural unit only responds to the area within the receptive field and does not care about the area outside the receptive field at all. Such local connectivity patterns ensure that the learned convolution kernels have the strongest response to the input spatial local patterns. The weight-sharing network structure makes it more similar to the biological neural network, which reduces the complexity of the network model and the number of weights. This network structure is highly invariant to translation, scaling, tilting, or other forms of deformation. Moreover, the convolutional neural network uses the original image as input, which can effectively learn the corresponding features from a large number of samples, avoiding the complex feature extraction process.

In our approach, we introduce a convolutional neural network model to classify and identify the extracted feature vector. Given the feature vector *F*, the classification process can be described in the following:

(8) $$\begin{array}{c} \text{Result}=M\left(F,\theta \right), \end{array}$$

where the *M*(·) represents the mapping function whose network model parameter is *θ*. The model takes *F* as input and outputs the classification result Result. Based on that, we adopt the cross entropy as loss function to optimize the model. The definition is as follows:

(9) $$\begin{array}{c} \theta^{*}=\underset{\theta }{\text{argmin}}L\left(\theta \right)=\underset{\theta }{\text{argmin}}-\sum_{i\in \Lambda }\sum_{c}q_{i}\left(c\right)\text{ln}\left(P_{i}\left(c\right)\right), \end{array}$$

where *q*_*i*_ is the one-hot vector corresponding to the label *y*_*i*_, and *q*_*i*_ ∈ **R**^*C*^, ‖*q*_*i*_‖_1_=1, *q*_*i*_(*c*) ∈ {0,1}, *q*_*i*_(*y*_*i*_)=1. For the C classification problem, record the output of the prediction node as *z*_*i*_(*c*), *c*=0,…, *C* − 1; then, the predicted probability obtained by the softmax function is

(10) $$\begin{array}{c} P_{i}\left(c\right)=\frac{e^{z_{i}\left(c\right)}}{\sum_{m=0}^{c-1}e^{z_{i}\left(m\right)}}. \end{array}$$

Calculate the derivative of the loss function *L*(*θ*) with respect to *z*_*i*_(*c*) as

(11) $$\begin{array}{c} \frac{\partial L}{\partial z_{i}\left(c\right)}=P_{i}\left(c\right)-q_{i}\left(c\right). \end{array}$$

Then, the network weights can be updated according to the loss backpropagation algorithm. The whole constructure of the network is shown in Figure 3. The training algorithm of the classifier is shown in Algorithm 2.

## 3. Experiments and Results

In this section, in order to verify the effectiveness of the above methods, we use Human Activity Recognition Using Smartphones Dataset to conduct sufficient experiments, including classification performance analysis, effectiveness analysis of feature processing methods, and comparison with current state-of-the-art processing methods.

### 3.1. Data Description and Metrics

We utilized the Human Activity Recognition Using Smartphones Dataset [21] to evaluate our proposed method in our experiments. The Human Activity Recognition Dataset was constructed by some experiments. The experiments have been carried out with a group of 30 volunteers within an age bracket of 19–48 years. Each person performed six activities wearing a smartphone (Samsung Galaxy S II) on the waist, including walking, walking upstairs, walking downstairs, sitting, standing, and lying. Using its embedded accelerometer and gyroscope, the wearable device captured 3-axial linear acceleration and 3-axial angular velocity at a constant rate of 50 Hz. The sensor signals (accelerometer and gyroscope) were preprocessed by applying noise filters and then sampled in fixed-width sliding windows of 2.56 sec and 50% overlap (128 readings/window). The sensor acceleration signal, which has gravitational and body motion components, was separated using a Butterworth low-pass filter into body acceleration and gravity. The gravitational force is assumed to have only low-frequency components; therefore, a filter with 0.3 Hz cutoff frequency was used. From each window, a vector of features was obtained by calculating variables from the time and frequency domains. The experiments have been video-recorded to label the data manually.

The obtained dataset has been randomly partitioned into two sets, where 70% of the volunteers were selected for generating the training data and 30% were selected for generating the test data. For each record in the dataset, it contains the triaxial acceleration from the accelerometer, the estimated body acceleration, the triaxial angular velocity from the gyroscope, a 561-feature vector with time and frequency domain variables, and the activity label. In the dataset, there are six types of human activities, including walking, walking upstairs, walking downstairs, sitting, standing, and lying. Each type of data has been divided into training dataset and testing dataset in the original database as shown in Table 2, and thus we utilized them directly without further data division.

In our method, we adopt an intelligent data processing method based on deep learning technology. In order to better adapt to the learning characteristics of the neural network, the following normalized preprocessing methods are adopted before feature extraction of data:

(12) $$\begin{array}{c} x_{\text{min}-\text{max}}=\frac{x-x_{\text{min}}}{x_{\text{max}}-x_{\text{min}}},\\ x_{\text{zero}}=\frac{x-\bar{x}}{\sigma }. \end{array}$$

The first data preprocessing method can normalize the data values to the range of 0 to 1, which is more conducive to the training and learning of neural networks. The second normalization method normalized the original dataset into a dataset with a mean of 0 and variance of 1, so that the features of the dataset could be learned more easily by the neural network model.

We use the following famous metrics to evaluate the experimental performance: accuracy (Acc), sensitivity (Sen), specificity (Spe), and positive predictive value (PPV). Their definitions are given as follows:

(13) $$\begin{array}{c} \text{Acc}=\frac{\text{TP}+\text{TN}}{\text{TP}+\text{TN}+\text{FP}+\text{FN}},\\ \text{Sen}=\frac{\text{TP}}{\text{TP}+\text{FN}},\\ \text{Spe}=\frac{\text{TN}}{\text{TN}+\text{FP}},\\ \text{PPV}=\frac{\text{TP}}{\text{TP}+\text{FP}}, \end{array}$$

where TP is the number of true positive detections, TN is the number of true negative detections, FN represents the number of false negative detections, and FP represents the number of false positive detections.

### 3.2. Feature Analysis

In order to verify the effectiveness of feature extraction designed in the method, a comprehensive analysis was performed in the experiment. We compared the results in the following four cases:

- Condition 1: process the data only with the statistical methods.
- Condition 2: process the data only with the autoencoder model methods.
- Condition 3: classify the data with the convolutional neural network model methods.
- Condition 4: classify the data with the SVM methods.
- Condition 5: use the proposed method to process and classify the data.

Table 3 describes the results produced under the five data processing and classification scenarios described above. It can be seen that the classification results are the worst when using the convolutional neural network or SVM classifier alone to classify the data. When the data are processed by statistical methods or autoencoders, the classification results will be improved to a certain extent, which shows that these data processing methods can effectively extract features from the data. Our proposed method combines statistical methods and feature extraction methods from autoencoders, which achieves the best results and also demonstrates the effectiveness of our method.

At the same time, we compared the results of the ablation experiments for each calculation method in the statistical method. The experimental results are shown in the histogram in Figure 4. It can be seen that the role of frequency-domain features is slightly larger than that of the time-domain features.

### 3.3. Comparison with Other Methods

This experiment compares the existing advanced intelligent sports training data processing methods, including CNN, SVM, multi-class SVM [22], and Convnet method [23].  Table 4 describes the results of each method under the four metrics, including accuracy (Acc), sensitivity (Sen), specificity (Spe), and positive predictive value (PPV). As can be seen from Table 4, our proposed method achieves the best classification results, which demonstrates the effectiveness of the wearable device-based smart sports training data processing method proposed in this paper.  Figure 5 shows the confusion matrix of the average classification results, and it can be seen that the classification performance of each category has reached more than 90%, which fully proves the effectiveness of our proposed method.

## 4. Conclusion

Physical training is an important item of basic physical fitness and skill training. Deeply excavating the inherent characteristics of physical training data and identifying sports types can optimize the implementation of physical training guidance and effectively improve the effect of physical training. The application of deep learning in the field of sports simplifies the processing of massive data and people have a new understanding of the data in the field of sports, which will play a positive role in promoting the further application of deep learning in the field of sports in the future. This paper proposes an intelligent processing method for sports training data processing, which integrates statistical methods and deep learning techniques to extract the intrinsic features in the original data, so as to be able to identify different types of sports. In future, a practical experiment platform will be built. In addition, more application-based wearable devices will be considered.

## Figures and Tables

**Figure 1:** The overall flowchart of the proposed method.

**Figure 2:** The autoencoder model designed in our approach.

**Figure 3:** The convolutional neural network model.

**Figure 4:** The effect of each feature on the classification accuracy in the ablation experiment.

**Figure 5:** The confusion matrix of the average classification results.

**Algorithm 1:** The training algorithm of the autoencoder.

**Algorithm 2:** The training algorithm of the classifier.

**Table 1:** The statistical methods used in the data preprocessing.

Type	Name	Equation
Time domain	Mean	$\bar{X}=1/n\sum_{i=1}^{n}X_{i}$
	Variance	$s^{2}=\sum_{i=1}^{n}{\left(X_{i}-\bar{X}\right)}^{2}/n$
	Kurtosis	$K=\sum_{i=1}^{n}{\left(X_{i}-\bar{X}\right)}^{4}f_{i}/ns^{4}$
	Covariance	$\text{cov}\left(X,Y\right)=\sum_{i=1}^{n}\left(X_{i}-\bar{X}\right)\left(Y_{i}-\bar{Y}\right)/n-1$
	Skewness	$\text{S}K=n\sum_{i=1}^{n}{\left(X_{i}-\bar{X}\right)}^{3}/\left(n-1\right)\left(n-2\right)s^{3}$
	Correlation coefficient	$i_{xy}=\sum_{i-1}^{n}\left(X_{i}-\bar{X}\right)\left(Y_{i}-\bar{Y}\right)/\sqrt{\sum_{i=1}^{n}{\left(X_{i}-\bar{X}\right)}^{2}\sqrt{\sum_{i=1}^{n}{\left(Y_{i}-\bar{Y}\right)}^{2}}}$

Frequency domain	Entropy	*H*(*X*)=−∑_*k*=1_^*N*^*X*_*i*_(*k*)log*X*_*i*_(*k*)
	Energy	*E*=∑_*k*=1_^*N*^*X*_*i*_(*k*)^2^/*N*, (*X*_*i*_(*k*)=∑_*n*=1_^*N*^*x*_*i*_*e*^−*j*2*πkn*/*N*^, *k*=1,2,3,…, *N*)

**Table 2:** The data division used in our experiments.

Type	All samples	Training samples	Testing samples
Walking	1722	1226	496
Walking upstairs	1544	1073	471
Walking downstairs	1406	986	420
Sitting	1777	1286	491
Standing	1906	1374	532
Lying	1944	1407	537

**Table 3:** The result comparison under different conditions.

Condition	Acc (%)	Sen (%)	Spe (%)	PPV (%)
Condition 1	90.42	90.8	89.32	89.74
Condition 2	92.3	91.46	92.48	88.29
Condition 3	86.16	87.49	90.43	87.31
Condition 4	83.23	85.42	83.19	86.47
Condition 5	**95.62**	**95.21**	**98.17**	**96.65**

**Table 4:** Comparison with other methods.

Method	Acc (%)	Sen (%)	Spe (%)	PPV (%)
CNN	86.16	87.49	90.43	87.31
SVM	83.23	85.42	83.19	86.47
Multi-SVM [22]	88.97	89.35	97.66	89.23
Convnet [23]	94.5	94.79	**98.86**	94.78
Ours	**95.62**	**95.21**	98.17	**96.65**

## Data Availability

The data used to support the findings of the study are included within the article.
